RETRACTED

# Automation of Cephalometrics Using Machine Learning Methods

**DOI:** 10.1155/2022/3061154

**Published:** 2022-06-21

**Authors:** Khalaf Alshamrani, Hassan Alshamrani, F. F. Alqahtani, Ali H. Alshehri

**Affiliations:** Radiological Sciences Department, College of Applied Medical Sciences, Najran University, Najran, Saudi Arabia

## Abstract

Cephalometry is a medical test that can detect teeth, skeleton, or appearance problems. In this scenario, the patient's lateral radiograph of the face was utilised to construct a tracing from the tracing of lines on the lateral radiograph of the face of the soft and hard structures (skin and bone, respectively). Certain cephalometric locations and characteristic lines and angles are indicated after the tracing is completed to do the real examination. In this unique study, it is proposed that machine learning models be employed to create cephalometry. These models can recognise cephalometric locations in X-ray images, allowing the study's computing procedure to be completed faster. To correlate a probability map with an input image, they combine an Autoencoder architecture with convolutional neural networks and Inception layers. These innovative architectures were demonstrated. When many models were compared, it was observed that they all performed admirably in this task.

## 1. Introduction

The difficulty of defining characteristic points (detailed for each topic) in medicine is crucial since it improves the precision and speed of various medical examinations, ultimately helping patients. These studies used quantitative cephalometry. Cephalometric study determines the size and position of the teeth, jaws, and skull. This analysis aids in therapy planning, treatment evaluation, and clinical research. Cerebral cephalograms can be difficult to read. An X-ray shows the skull as a single 2D projection of a 3D entity, with overlapping components. Face asymmetry, head orientation, and radiography distortion all generate duplicate structures. Individual anatomical diversity and pathological circumstances make it difficult to assign cephalometric points consistently [1, 2]. Locating cephalometric spots on lateral cephalograms is difficult. Because an X-ray shows the skull as a 2D plane, the various structures appear to overlap. Duplicate structures emerge from facial asymmetry, head movement variations during photo acquisition, and radiographic distortion. Cephalometric points are difficult to locate precisely due to anatomical variance, especially in sick states. These areas are now recognised manually or semi-automatically, causing inconsistencies between orthodontists (inter-orthodontist mistakes) and among orthodontic practitioners (intra-orthodontist errors). Inter- and intra-observer variability may be affected by orthodontic training and experience [8, 9]. Also, time constraints and other commitments are considered. Convolutional networks (CNNs), occupying state of the art for various tasks in computer vision, have proven to be successful for a wide range of applications, including image classification [14, 18], image segmentation, the alignment of images [16], the detection of facial points [4], the estimation of human postures [21], and the detection of lines on roads [11, 12], among other tasks. Currently, it is in the field of medicine that a great trend has been seen in the use of CNN to automate the process of detecting and diagnosing diseases [6, 17, 7, 5].

RETRACTED

Using software that assists or advises the expert in marking the cephalometric points is one technique to optimise the process. This programme does not replace the need for a professional but rather gives tools to make your job easier. One example is CefMed, which allows all cephalometric point marking to be done from its platform, without needing the patient's X-ray image in physical format. This problem has no fully automatic or precise solution; hence, it has become a recent subject of scientific investigation. Currently, public and labelled databases (previously analysed by experts) are available, making it simple to research, develop, and compare studies. Ibragimov et al. [13] proposed a game theory and random forest solution. Using convolutional neural networks to detect cephalometric points, Arik et al. 2017 [3] merged a probability map of the cephalometric points based on the intensity of the pixels with a random forest model to construct a map based on the distribution of each point relative to the rest. This proposal outperformed the models offered by 2 mm, which is regarded as acceptable in dentistry. Juan Ignacio Porta [20] proposed a new architecture that uses a CNN with Inception layers and an Autoencoder to assign a probability map to an image input. The goal is to generate Bjork–Jarabak and Ricketts cephalometrics automatically.

## 2. Methodology

To carry out a supervised learning model, it is necessary to have labelled information; the only available information was the public dataset of the competition “Grand Challenges in Dental *X*-ray Image Analysis. Challenge #1: Automated Detection and Analysis for Diagnosis in Cephalometric *X*-ray Image.” The dataset comprises a training set of 150 images and 2 evaluation sets of 100 and 150 images, respectively. It contains images of patients between 6 and 60 years old, and contains nineteen of the most popular cephalometric points as reference points to detect. The original image sizes are 2400 × 1935 pixels, and the resolution is 0.1 mm/pixels in both directions. The images were compressed to one third of the original image (taking the average of each 3 × 3 patch) for dimensionality reduction purposes; this reduces the computational complexity without losing important information, resulting in an 800 × 645 image. The nineteen dataset points do not make up any specific cephalogram.

RETRACTED

For this reason, it is not possible to train a machine learning model that detects all points in a cephalogram. However, it is useful to be able to check the performance of the model and to be able to compare it with other existing models in the literature. To solve this problem, it was necessary to create a dataset containing information on the cephalometric points of each of the different cephalograms, Bjork–Jarabak and Ricketts in this case.

### 2.1. Creating a Dataset

It was feasible to collect tagged photos of several types of cephalograms by collaborating with the company CefMed. With these data, a machine learning model could ideally be created to detect and label X-ray pictures for each type of cephalogram automatically. Several issues were discovered after the data was analysed:

1. The X-ray images had different sizes (different aspect ratios) and resolutions (mm/pixels)
2. The images were neither not taken with the same equipment, nor by the same operators
3. Some images were not originally digital and some digitisation processes had been applied to them, such as scanning or directly taking a photograph, either on a monitor or a negatoscope
4. The images did not have the same levels of contrast and brightness
5. The images were labelled by different professionals.

Considering these and other issues, creating a dataset is not easy. A solution had to be found for each issue. As stated previously, the photos were tagged by experts. Experiment 1 shows a range of 0.4 mm to 3.7 mm (SD = 0.2–2.5 mm) for the same examiner, and 0.6 to 5.3 mm (SD = 0.2–3.2 mm) for different examiners. A cephalogram has a tolerance of 2 mm, according to experts. So a point can be found within 2 mm of its actual distance and the cephalometric readings are still valid. Creating a dataset with data from multiple specialists would increase the variance in each point's label, making the process more challenging. As a result, each dataset has data from a single physician. The data has to be normalised to match the photos' brightness and contrast levels (some images were RGB with bluish tints). Because the photos had varying aspect ratios, it was required to devise a process to crop them while keeping their information. To achieve this, two methods were used: binarize the crop and use supplementary information to detect the target area.

RETRACTED

#### 2.1.1. Cropping Images Using Binarisation

Aspect ratio cropping was required after obtaining the photos. For starters, the image's centroid is calculated. So, photos having a threshold were binarised, i.e., values below the threshold were assigned 0 and above the threshold were allocated 1. A box with a fixed aspect ratio is placed in that spot according to the existing convolutional model input, 800px × 600px, using this information. So, when using the box to crop, certain areas were outside the image and had to be filled in with supplementary information (Figure 1). We used zeros, average image value, and constant values along the image's edges. As a result, the images produced by this method were cluttered and noisy.

#### 2.1.2. Cropping Images Using Soft Structure

Seeing as the previous approach did not work, it was decided to find a new way to crop photographs more efficiently and use all the extra information available from each image. Each one is marked with the cephalometric points and the soft and hard profiles of the X-ray images of the skin and bones. We can determine where the region of interest is on the original image using this data.

Each structure's data was represented as a set of points, which were then interpolated to produce a line with coordinates (*x*, *y*). This was done for each image, saving the measurements of each box. Then, a statistical analysis was done to produce a box with average measurements. This served two purposes: First, an exploratory study of the data to get a sense of the photos accessible. Second, to get the trimmed photos' aspect ratio. Using the data, it was concluded that the photos' aspect ratio diverged from the Challenge dataset. So, a box (790Px × 653Px) was created to match the Challenge magnets. The steps were as follows: To locate the box, a raw image was acquired first, with all the points (cephalometric and structural) recognised. If the box is too tiny, it is enlarged while keeping the same aspect ratio, increasing equally on each side until all points are within it. The image is ready to utilise after the box is determined. It must be compressed to use a larger box, but because it has the same aspect ratio as our model input; this can be done without distorting the image.  Figure 1(d) depicts the above method. The box in blue will be used to crop the image (it needs to be expanded due to the image dimensions). Before using this cropped image, it must be reduced to (790 × 653). The (*x*, *y*) coordinates are distinct and utilised to check the coloured lines for hard and soft tissue features. The box points are good.

RETRACTED

### 2.2. Inception Layers

There is a simple yet powerful approach to improving deep learning models. You can simply construct a larger model, either in-depth, i.e. number of layers, or neurons per layer. But, as you might expect, it can cause problems: overfitting is more likely to occur with larger models, especially when training data is limited. Increasing the number of parameters means increasing computational resources. Assume, for example, that a layer in our deep learning model has learned to focus on specific features of a face (Figure 2). The following layer of the network would probably focus on the image's public face to identify the things there. The layer must have the necessary filter widths to identify various objects to do this. Figures 2(b) and 2(c) show that X-ray structures are modest and vary in size depending on age, race, etc.

The age difference affects the size of the structures. The Inception layer [22] stands here. It allows the inner layers to search and select the appropriate filter size. So, even if the size of the structures in the image varies, like in Figures 2(d) and 2(e), the layer works to recognise the structures. I would probably use a larger filter size for the first image and a smaller one for the second. A larger filter is chosen for global information, whereas a smaller filter is preferred for local information. Various iterations of the Inception layers were shown throughout time. The InceptionD and InceptionE layers were employed here. As a result, employing these layers in convolutional networks is computationally expensive. So, the number of filters in each layer was reduced, resulting in lighter versions. Figures 3 and 4 show the adjustments implemented.

### 2.3. Autoencoder

An Autoencoder is a form of unsupervised artificial neural network used to learn efficient data encodings.  Figure 5 shows an autoencoder's structure. It has two components: encoder and decoder. To reduce the dimensionality of a data collection, an encoder learns an encoding by training the network to disregard “noise” in the signal. Along with the reduction side, the network learns a reconstruction side, the decoder, where it tries to recreate the input from encoding as closely as feasible. By way of example, an X-ray image can be learned to encode basic properties like corners or edges, then parsed and encoded by subsequent layers. Decoder layers learn to decode representations to rebuild the original input image.

Below is an Autoencoder with Inception layer design. The input image is 800 × 645 according to the dataset utilised. This is followed by an image of how it was updated to work with various datasets.  Figure 6(a) depicts the encoder architecture. A normalising layer and a ReLU as an activation function follow each 2-D convolution layer. Stride 2 for the first layer 1 for the next two. Only one of the three 2-D convolutions has a padding of 1. After the 2-D convolution layer comes to a maxpooling layer with two kernel. Three Inception layers follow. 1 InceptionD, 2 InceptionE. The encoder outputs a 98 × 79 image (approximately 8x dimensionality reduction).  Figure 6(b) shows the decoder design with five layers of 2-D transposed convolutions, the first and fourth with a Stride of 1, and the rest with a Stride of 2. The Autoencoder's output is sigmoid functioned to get a scalar in the interval (0, 1).

RETRACTED

### 2.4. Probability Maps

As previously stated, autoencoders can be used to reconstruct network input data. So, an Autoencoder cannot directly recognise cephalometric points in an image. We can train the model to find spots within an image. Activation maps were created for each cephalometric point using each image's coordinates (*x*, *y*). To detect the position of the Landmark, a Gaussian function with a maximum inaccuracy of 2 mm is centred in those regions where the probability maps are formed. Figures 7(a)–7(d) show the outcome of this operation. The ISBI dataset images of 800 × 645 would result in a collection of activation maps of the type (19, 800, 645), one for each cephalometric point. An Autoencoder can be trained to recreate this information using these activation maps and the original image. The autoencoder learns to build activation maps for each point during this process, with the highest activation areas predicting the point's coordinates.

#### 2.4.1. Cost Function

To fit a function whose image belongs to Rn, models like Autoencoders are used. This would suggest that the suitable cost function is the Mean Square Error, which is frequent in regression situations, but because our output is unique, our model's image is [0, 1] *n* Rn and we are. Since we are comparing probability distributions, the binary cross entropy is a good fit. The cost function incorporates the Sigmoid output to improve numerical stability, and the positive class can be weighed to trade recall for precision.

#### 2.4.2. Inception Autoencoder with the New Dataset

Changes were made to the structure of the Inception Autoencoder based on the dataset created. The new architecture receives images of (790Px × 653Px). As for the output, we only have 7 (and 36 respectively) output layers depending on the type of Ceph we are trying to predict.

### 2.5. Preliminary Tests

The next section details many preliminary tests conducted to understand the problem better and explore possible solutions. The first experiment used the Autoencoder Inception 2.4.2 architecture but doubled the number of filters in the decoder's convolutional layers. Because the encoder had the most trainable parameters, the objective was to balance the number of parameters across the architecture. They were assured that both portions of the architecture could learn the task for which they were educated.  Figure 8 shows the revised decoder architecture.

RETRACTED

In both experiments, Autoencoder Inception 2.4.2 was used as the basic architecture. In the decoder, more convolutional layers were added to the model to balance the number of trainable parameters.

#### 2.5.1. Menpo

The third experiment used an image alignment model. An active appearance Model is a deformable statistical model of an object's shape and appearance. It uses an optimisation approach to get a parametric description of an object during training. The cephalometric points from the training images were used to construct a model. The AAM was designed to help the autoencoder make more precise predictions since it has more spatial information between the cephalometric points. In this experiment, an AAM trained on cephalometric points was applied to the underlying architecture of the autoencoder Inception 2.4.2. So, the AAM creates new predictions, also in coordinate form. This experiment uses the Menpo library, which offers 2D and 3D deformable modelling tools.

#### 2.5.2. Shape Model

For the fourth experiment, Ibragimov et al. presented a game-theoretic framework for segmenting images based on reference points. In this game, the landmarks are players, the candidate points are strategies, and the probabilities that the candidate points represent a candidates in the target image are compared to landmarks in images from the training set to determine if they are similar in image. The highest *n* activations of a probability map were used as candidate points to solve an optimisation problem based on game theory. However, the computational cost of solving this problem prevented extensive testing, so this idea was abandoned.

#### 2.5.3. Various Activation Functions

Various autoencoder activation functions were tried. Leaky ReLU and PReLU were chosen. The reason for using Leaky ReLU is that it avoids the problem of null activations when the neuron value is less than 0, which prevents learning in ReLU. PReLU is based on Leaky ReLU and has less accuracy than ReLU. Unlike Leaky ReLU, PReLU uses a parameter instead of 0.01.

### 2.6. Proposed Models

The next section describes the changes made to the original model. First, Xavier's idea changed the initialisation of the convolutional layer weights [10]. Xavier initialisation in neural networks avoids starting activation functions in saturated or dead regions. Or, we want to set the weights to values that are “just right.” Xavier initialises a layer's weights using a random uniform distribution, where *ni* is the number of connections entering the layer and *ni* + 1 is the number of connections leaving it.

RETRACTED

#### 2.6.1. Wider Model

The second change widened the convolutional layers' receptive field. The receptive field is the region in the input space from which a CNN feature can obtain information. The size of the convolutional layer kernels was changed, and an Inception layer was added to the encoder.  Figure 9 shows the new architecture. The changes made to the architecture are detailed below: encoder's first convolutional layer's kernel size increased. It went from 3 × 3 to 5 × 5, with 2 paddings. The encoder's second layer now includes Inception E. Change the number of filters in subsequent layers to add a convolutional layer to smooth the dimensionality decrease.

#### 2.6.2. Wider Paddup Model

The third change made to the model was how the decoder reconstructs the “image” (probability map). Checkerboard artefacts in the output images are the most common issue with transposed convolution. So, the transposed convolutional layers were replaced by upsampling with basic convolutions, as in [19]. The following convolutional layers were transposed: the probability map is first upscaled using nearest-neighbour, then constant padding, and finally convolution.

#### 2.6.3. Gray Models

The fourth modification involved changing the structure to accept grayscale images. This was done because the model was trained on RGB images containing irrelevant information. So, we added a grayscale transformation and reduced the number of input channels from 3 (RGB) to 1 (grayscale). This change was made to the original model and the experiments mentioned in this section to see if their performance changed. The transformation averages the three channels, as shown in Figure 9.

### 2.7. Models with Extra Point Information

The fifth experiment used extra image data to improve the model. This data was used to create new probability maps based on the locations of the soft and hard profiles. The points are easier to identify because they are all marked on some profile (soft or hard). In the beginning, experts found it difficult to locate information from the mandible, Silla, and Basion areas. They were created using the same criteria as the cephalometric points. Previously, a structure's line or trace had to be interpolated between points and then mapped using Gaussian functions. The original points for both structures are on the left, and the result is on the right. Adding two probability maps (one for each structure) added two more input layers. This test used autoencoder wider.

RETRACTED

#### 2.7.1. Box to Find Activations

The sixth experiment attempted to resolve one of the models' flaws: positive activations in areas where no cephalometric points could be found. Each dataset used the training data to calculate an average area for each point to solve this. These areas were calculated to other points (which the network correctly detects) to improve prediction accuracy for an unknown image. For each point, a box with the average distances to Pogonio and Silla points is set up, and the size of the box is determined by the training set's shortest and largest distances (plus a certain margin of error). The Silla point is green, while the Nasion and PiC points are orange. Red indicates the distance between the Silla point and PiC, and blue signifies the distance between the Silla point and the Nasion point. Using the same idea to avoid false detections for the Pogonio and Silla points was proposed. To do so, the average *X* and *Y* coordinates of their locations were calculated using the training data, and the same procedure was used for the rest of the cephalometric points [15].  Figure 10 shows a test image with two high probability zones for the Gonion point, one correct and one false. This method ignores false activation and calculates the prediction on the appropriate zone.

#### 2.7.2. Skeletonization and Tangent

It is a thin version of the shape equidistant from its boundaries. The skeleton emphasises the shape's connectivity, topology, length, direction, and width. Skeletonization results from thinning, which reduces the object's contour to an average of one pixel. An algorithm that calculates a skeleton from an image of a letter. A skeleton is a primitive object used in computer vision, image analysis, pattern recognition, and digital image processing. To find the Gonion (Go) point, two straight lines intersected, one armed with the articular and inferior poster points of the mandible ramus (PiR), the other with the Mentonian point and the lower posterior of the body (PiC). The PiR and PiC are difficult to mark, even for experts, causing errors in the lines and propagating the error towards the Gonion point. The PiR and PiC points (Figures 11(a) and 11(c)) were skeletonised in an experiment (Figures 11(b) and 11(d)). After obtaining the zone skeletons, both points were detected using the cephalometric rules.

#### 2.7.3. CordConv Model

It was proposed by Rosanne Liu et al. Using extra coordinate channels, the proposed solution, CoordConv, allows the fonvolution to access its input coordinates. The proposed CoordConv layer extends the standard convolutional layer by concatenating additional channels filled with coordinate information (i.e., constant information that is not trained). So, for example, a matrix with the first row 0 and the second row 1 is a coordinate channel *i*. The coordinate channel *j* is similar, but it has columns of constant values instead of rows. Two CoordConv layers were added to the Autoencoder Wider PaddUp architecture in this experiment, one for the encoder and one for the decoder.

RETRACTED

## 3. Experiments

Autoencoder Xavier, Autoencoder Wider, Autoencoder Wider Paddup, and Autoencoder Cord Conv were the models proposed in this work. On these models, various variations were tested, including Gray (grayscale images), Points (information on skull structures), Box, and Skeletonization. It is important to note that the following results are the first to be presented on private datasets and with real use cases when writing this special undergraduate project. This is significant because it allows us to see how these models are developed in practice. While competition results can provide metrics and results, nothing guarantees that the same results will be achieved in practice when developing a system that works with some of the aforementioned architectures. The training problem is presented in the first section, while the evaluation stage of each model is addressed in the second.

### 3.1. Landmark Selection from Probability Maps

Once the probability maps have been generated, it is necessary to establish some technique to determine only the position of each cephalometric point. A simple methodology was chosen, applying a Gaussian filter to the probability map (to filter possible false detections with high probabilities in particular areas) and choosing the point of greatest activation after the filter. The parameter *σ* of the Gaussian filter was chosen with the same restrictions imposed by the problem, that is, to detect a maximum error of 2 mm.

### 3.2. Hardware and Software Used

During the entire development process, a server provided by the High Performance Computing Center of the National University of Córdoba and the training and testing of the different proposed models were used. The server specifications are as follows:

1. Nebuchadnezzar Computer
2. Supermicro 1027GR-TSF node with X9DRG-HF motherboard
3. 2 Xeon E5-2680v2 of 10 cores each
4. 64 GiB RAM on 8 × 8 GiB DDR3 1600 MT/s modules
5. 3 NVIDIA GTX 1080Ti GPUs (GP102, 11 GiB GDDR5) connected by PCIe 3.016x
6. 1 SSD 240GiB for Operating System connected to SATA-2
7. 3 SSD 1TiB for data in RAID0 by ZFS connected to SATA-3.

RETRACTED

Software versions used:

1. Python 3.7
2. PyTorch 1.1.0
3. OpenCV 4.1.0.

### 3.3. Training

#### 3.3.1. Transformations on the Dataset

Before training the models, transformations are performed on the dataset, each one with a specific objective. In all the Autoencoder models developed, in addition to the reduction of the image mentioned in Section 3.1, a series of transformations are carried out to increase the amount of data that the model observes in the training phase, they are as follows:

1. Random image rescaling (between 98% and 102%)
2. Horizontal and vertical random translations to the image (up to 2% of the image in each direction)
3. Random image rotations (up to 5°)
4. Normalisation of the set of images to have mean 0 and variance 1.

The changes of scale, rotation, and random translation of the images are made at the beginning of each training epoch to artificially increase the size of the training set and thus achieve that the model better appreciates the existing structures in the images. The values chosen are values consistent with natural variations in the generation of the radiograph. These values are small because the cephalometric radiographs must be performed with a series of precautions that do not allow too much variation. The normalisation of the dataset is done to facilitate learning since there is no preferential dimension in the presented scale.

#### 3.3.2. Hyperparameters

In this section, we will determine the values of the model hyperparameters such as the learning rate ǫ, the regularisation weight *λ*, the weight of the positive class *p*, the batch size, and the number of learning epochs. A grid search similar to that of [20] was performed. The values obtained were: ǫ of 10^−3^, *λ* of 10^−5^, and *p* of 2500. The number of learning epochs was set to 300 epochs, and the batch size was modified on a per-experiment basis due to GPU memory constraints.

#### 3.3.3. Evaluation Sets

For the ISBI dataset, there are two evaluation sets, with 150 and 100 images, respectively. With the data provided by the company CefMed, 5 datasets were created following the strategies above, each with its respective subset for training and testing. The sets were assembled in such a way that each one of them was labelled by a different professional; the result of this was that the images of each set came from different medical centres, which meant a difference in resolutions, aspect ratios, colors, etc. Sets 1, 2, and 3 are from Bjork cephalometrics, set 4 is formed by the union of Sets 2 and 3, and set 5 are from Ricketts cephalograms.

### 3.4. Metrics

#### 3.4.1. Coefficient of Successful Detections

Instead of marking an area, the doctors mark the location of a single-pixel for each landmark. The detection is considered successful if the absolute difference between the detected and reference points is less than *z* mm. Otherwise, the detection is deemed unsuccessful. Then, with precision less than *z* mm, the coefficient of successful detections [26] (SDR for short) *Pz* is formulated as

(1) $$\begin{array}{c} p_{z}=\frac{\#\left\{j:\left\|L_{d}\left(j\right)-L_{r}\left(j\right)\right\|<z\right.}{\#\Omega }\times 100\%\ldots , \end{array}$$

where *L*_*d*_, *L*_*r*_ represent the location of the detected landmark and the labelled landmark, respectively, *z* denotes the measurement precision, in our case *z* = 2 mm due to the restrictions of the problem, although values such as 2, 5 mm, 3 mm, and 4 mm; *j* Ω, and #Ω represents the number of detections made. An important clarification is that to calculate the metric correctly, the different resolutions of each image must be taken into account, that is, the pixel/mm ratio of each one.

RETRACTED

#### 3.4.2. Mean Radius Error

The radial error [26] is defined as $R\;=\;\sqrt{\Delta x^{2}\;+\;\Delta y^{2}}$, where ∆x, ∆y is the absolute distances in the *x* and *y* directions, respectively, between the detected landmark and labelling. The mean radial error or mean radial error (MRE) and the associated standard deviation or standard deviation (SD) are calculated.

## 4. Results and Discussion

This section will present the results of the different experiments presented in section 3.6. For each experiment, a dataset was chosen on which to train the models. The success detection rate is calculated as an average for the 7 (or 36) cephalometric points in the following graphs. The models were trained for 300 epochs and the metrics were calculated every 10 epochs.

### 4.1. Basic Autoencoder

In the first experiment, it was carried out for all available datasets to obtain a baseline to compare the different experiments. It can be seen that the model has a similar behavior for these datasets. Around epoch 100 of training, the models suffer from overfitting; they overfit the training data, making it impossible to generalise the prediction task for validation images. The models reach an SDR of 0.65 on average for the 7 cephalometric points in their respective test sets. If we examine the metrics for each cephalometric point (Table 1), we see that the model can predict the location of many cephalometric points with high accuracy, but for points 4 and 5, it has a detection coefficient which is very low, making the average metric drop. Similar results are observed except for set 6 where the initial values are greater than the rest.

An important result to mention is the results observed in datasets 2 and 3 (Sections 4.2 and 4.3). In the test set 2, it was possible to obtain an SDR of 0.24 while in test set 3 one of 0.75, these representing the minimum and maximum values observed. A comparison was made between the models in their respective test sets. In addition, the results obtained on dataset 6, that is, on the public dataset of the ISBI Challenge, were analysed. The metric values are similar to those of datasets 1, 3, and 4. Something important to clarify is that the SDR values start with higher values than the rest and then normalise like the others.

RETRACTED

### 4.2. Xavier

The results obtained were similar and no improvement was obtained.

### 4.3. Wider Model

The basic model achieves a maximum SDR of 0.64 while the Wider model is 0.70. On the other hand, the same comparison but with dataset 3 obtained a maximum SDR of 0.75 for the basic model while the Wider model was 0.84.

### 4.4. Wider Paddup Model

No substantial improvements were observed with this experiment and the values obtained for both the SDR and MRE were similar to that of the Wider model. This model stood out in Set 2, achieving the best results obtained on this dataset. If we compare with the basic autoencoder, where we had an SDR of 0.24 in test, we have that the Wider Paddup model achieves maximum values of 0.76.

### 4.5. Wider Gray Model

The Wider model's experiment of adding grayscale images was performed. No substantial improvements were observed with this experiment, and the values obtained for both the SDR and MRE were similar to the Wider model.

### 4.6. Points

The results obtained with the Autoencoder Wider Points model were compared, that is, the one that uses information from the skull structures, for the training set 2 against the best result obtained up to this point for that same set, that is, the Wider Paddup model. In addition, an experiment was carried out comparing the Autoencoder Wider Points model with a modified version that used grayscale images; the values obtained were similar, an SDR of 0.74 for the Wider Points model and one of 0.75 for the Wider Points Gray model.

### 4.7. Box

The experiment consisted of adding a box to locate the points restricting the search area for maximum activation on the Autoencoder Wider Paddup model. There were no significant changes for the SDR at 2 mm; however, the number of false predictions in areas where the points do not belong decreased. This can be observed for the metric values at 3 mm and 4 mm, which are not relevant due to the restrictions of the problem.

### 4.8. Box and Skeletonization

In the experiment of adding a box, the idea of using skeletonization was added to detect the points that had bad detections. The model improved the detection of these points but by a small margin (Table 2); this is observed in point 4, which improved the SDR by 10 points.

RETRACTED

### 4.9. Conv Coord

Finally, the performance of the Autoencoder Wider Paddup model was evaluated using Coord Conv layers. If we compare it with the version without these convolutional layers, we can notice a similar behaviour, concluding that no improvements were obtained.

## 5. Conclusions and Future Work

The dentist uses cephalometric analysis to diagnose dental, skeletal, and cosmetic issues. The majority of professionals do this manually, necessitating the development of tools. This study used machine learning to create cephalometry. The authors presented autoencoder-based Inception layers convolutional neural networks. The models detect specific points in images, especially cephalometric points on X-ray images. Despite the problem's constraints, they could detect cephalometric points at a 2 mm distance. Considerations: using high-resolution images and consistent X-ray equipment improves results. Multiple professionals labeling the same image is not allowed. To get accurate point data, you can have different dentists label all the images in a dataset. Less false activations and more localised probability maps resulted from adding extra information to the model, such as structure location.

More topics will be explored in this unique work in the future. Reducing intra-observer error requires more professionally labelled images in the dataset. This increases the model's image library and performance. This method can also be used in other fields of medicine, such as detecting tumours in X-ray images. The location data for the images' structures is a great addition to these models. Building cephalometrics or any other medical study that requires structure detection can benefit from investigating structure detection in X-ray images.

## Figures and Tables

**Figure 1:** RX Crop using centroids. (a) Original image, (b) thresholded image, (c) cropped image using average values to fill in the missing information. (d) Original image. In blue, a box is shown that covers all the points of the structures and where they will be cut. Each colored line represents a different structure.

**Figure 2:** (a) X-ray image extracted from the ISBI 2014 dataset. (b) 2X zoom of the original image; (c) 4X zoom of the original image; ((d), (e)) Two images from the dataset.

**Figure 3:** Modified InceptionD layer.

**Figure 4:** Modified InceptionE layer.

**Figure 5:** Diagram of the parts of an autoencoder.

**Figure 6:** (a) Architecture of an encoder with Inception layers. (b) Architecture of a decoder with Inception Inter2 layers.

RETRACTED

**Figure 7:** (a) Original image with the Silla point marked in red. (b) Heat map generated with a Gaussian activation centred on the coordinates of the point. (c) Original image with the Gonion point marked in red. (d) Heat map generated with a Gaussian activation centred on the coordinates of the point.

**Figure 8:** Autoencoder complex model decoder. The number of filters in all convolutional layers doubled.

**Figure 9:** Encoder architecture in the wider model. The size of the filters and padding have been modified and added one more Inception layer.

**Figure 10:** Transformation of images to grayscale. (a) Original image. (b) Image after transformation. (c, d) Calculation of box. In red distance between point Silla and PiC *X*-axis. In blue distance between point Silla and Nasion. (e) Original. (f) Image activation map of the convolutional model. (g) In blue, a rectangle calculated from the training data is observed. In red, a false detection outside the rectangle. (h) Image example with boxes and tan.

**Figure 11:** Skeleton.

**Table 1:** Coefficient of successful detections by landmark. Basic autoencoder model trained on Set 1.

	Training set				Test set			
	2 mm	2.5 mm	3 mm	4 mm	2 mm	2.5 mm	3 mm	4 mm
L1.00	0.96	0.98	1	1	0.85	0.9	0.93	0.93
L2.00	0.94	0.96	0.99	0.99	0.76	0.8	0.83	0.9
L3.00	0.98	0.99	1	1	0.76	0.76	0.8	0.9
L4.00	0.98	0.98	0.98	0.98	0.15	0.2	0.24	0.32
L5.00	0.7	0.79	0.85	0.91	0.29	0.44	0.46	0.51
L6.00	1	1	1	1	1	1	1	1
L7.00	0.95	0.97	0.98	0.98	0.66	0.71	0.8	0.83
Average	0.93	0.95	0.97	0.98	0.64	0.69	0.72	0.77

**Table 2:** Coefficient of successful detections by landmark. Model autoencoder wider Paddup box.

	Test box set				Skeletonization test set			
	2 mm	2.5 mm	3 mm	4 mm	2 mm	2.5 mm	3 mm	4 mm
L1.00	0.85	0.93	0.95	1	0.9	0.9	0.98	1
L2.00	0.8	0.88	0.9	0.98	0.83	0.9	0.93	0.98
L3.00	0.9	0.93	0.93	0.98	0.9	0.93	0.93	0.98
L4.00	0.27	0.29	0.39	0.44	0.37	0.39	0.39	0.51
L5.00	0.27	0.29	0.39	0.54	0.27	0.34	0.46	0.54
L6.00	0.95	1	1	1	0.98	1	1	1
L7.00	0.85	0.88	0.88	0.98	0.71	0.76	0.78	0.88
Average	0.7	0.74	0.78	0.84	0.71	0.75	0.78	0.84

## Data Availability

The data used to support the findings of this study are included within the article.

## References

[1] Kannan S. K. (2013). A simplified overview on clinical cephalometrics PJ Antony, S.karthiga Kanannan, Joby paulose, Manu M Mathew, Charis chandy joseph. *Journal of Indian Academy of Oral Medicine and Radiology*.

[2] Toman H. A., Nasir A., Hassan R., Hassan R. (2011). Skeletal, dentoalveolar, and soft tissue cephalometric measurements of Malay transfusion-dependent thalassaemia patients. *The European Journal of Orthodontics*.

RETRACTED

[3] Agrawal D. (2013). Cephalometric analysis for Diagnosis and treatment of orthodontic patients. *Journal of Oral Health and Community Dentistry*.

[4] Lee S. M., Kim H. P., Jeon K., Lee S.-H., Seo J. K. (2019). Automatic 3D cephalometric annotation system using shadowed 2D image-based machine learning. *Physics in Medicine and Biology*.

[5] Abdullah Hamad A., Thivagar M. L., Bader Alazzam M., Alassery F., Hajjej F., Shihab A. A. (2022). Applying dynamic systems to social media by using controlling stability. *Computational Intelligence and Neuroscience*.

[6] Song Y., Qiao X., Iwamoto Y., Chen Y.-W., Chen Y. (2021). An efficient deep learning based coarse-to-fine cephalometric landmark detection method. *IEICE - Transactions on Info and Systems*.

[7] Latif J., Xiao C., Imran A., Tu S. Medical imaging using machine learning and deep learning algorithms: a review.

[8] Sun J., Zhong G., Huang K., Dong J., Dong J. (2018). Banzhaf random forests: cooperative game theory based random forests with consistency. *Neural Networks*.

[9] Arik S. Ö, Ibragimov B., Xing L. (2017). Fully automated quantitative cephalometry using convolutional neural networks. *Journal of Medical Imaging*.

[10] Alazzam M. B., Al-Radaideh A. T., Binsaif N., AlGhamdi A. S., Rahman M. A. (2022). Advanced deep learning human herpes virus 6 (HHV-6) molecular detection in understanding human infertility. *Computational Intelligence and Neuroscience*.

[11] Kich I., Ameur E. B., Taouil Y. (2021). CNN auto-encoder network using dilated inception for image steganography. *International Journal of Fuzzy Logic and Intelligent Systems*.

[12] Barra P., Bisogni C., Nappi M., Ricciardi S. Fast QuadTree-based pose estimation for security applications using face biometrics.

[13] Bader Alazzam M., Mansour H., Hammam M. M. (2021). Machine learning of medical applications involving complicated proteins and genetic measurements. *Computational Intelligence and Neuroscience*.

[14] Zhang S., Huang W., Wang H. (2020). Crop disease monitoring and recognizing system by soft computing and image processing models. *Multimedia Tools and Applications*.

[15] Alazzam M. B., Mansour H., Alassery F., Almulihi A. (2021). Machine learning implementation of a diabetic patient monitoring system using interactive E-app. *Computational Intelligence and Neuroscience*.

[16] Novac P.-E., Hacene G., Pegatoquet A., Miramond B., Gripon V. (2021). Quantization and deployment of deep neural networks on microcontrollers. *Computer Science Machine Learning*.

[17] Mishra S., Stoller D., Benetos E., Sturm B., Dixon S. GAN-based generation and automatic selection of explanations for neural networks.

[18] Bach S., Binder A., Montavon G., Klauschen F., Müller K.-R., Samek W. (2015). On pixel-wise explanations for non-linear classifier decisions by layer-wise relevance propagationfier decisions by layer-wise relevance propagation. *PLoS One*.

RETRACTED

[19] Panda B. (2019). Hyperparameter tuning. *Project: Application of Population Based Algorithm on Hyperparameter Selection*.

[20] Alazzam M. B., Al-Radaideh A. T., Alhamarnah R. A., Alassery F., Hajjej F., Halasa A. (2021). A survey research on the willingness of gynecologists to employ mobile health applications. *Computational Intelligence and Neuroscience*.

[21] Atagün E. K. Y., Timuçin T., Gündüz H., Bayıroglu H. (2021). Effective factor detection in crowdfunding systems. *Trends in Data Engineering Methods for Intelligent Systems*.

[22] Zhao X., Xie C., Wang H. The research about containment the radial error propagation in self-servowriting in hard disk.

